# A Calibrated Multiexit Neural Network for Detecting Urothelial Cancer Cells

**DOI:** 10.1155/2021/5569458

**Published:** 2021-06-13

**Authors:** L. Lilli, E. Giarnieri, S. Scardapane

**Affiliations:** ^1^Department of Information Engineering, Electronics and Telecommunications (DIET), Sapienza University of Rome, Italy; ^2^Faculty of Medicine and Psychology, Sapienza University of Rome, Italy

## Abstract

Deep convolutional networks have become a powerful tool for medical imaging diagnostic. In pathology, most efforts have been focused in the subfield of histology, while cytopathology (which studies diagnostic tools at the cellular level) remains underexplored. In this paper, we propose a novel deep learning model for cancer detection from urinary cytopathology screening images. We leverage recent ideas from the field of multioutput neural networks to provide a model that can efficiently train even on small-scale datasets, such as those typically found in real-world scenarios. Additionally, we argue that calibration (i.e., providing confidence levels that are aligned with the ground truth probability of an event) has been a major shortcoming of prior works, and we experiment a number of techniques to provide a well-calibrated model. We evaluate the proposed algorithm on a novel dataset, and we show that the combination of focal loss, multiple outputs, and temperature scaling provides a model that is significantly more accurate and calibrated than a baseline deep convolutional network.

## 1. Introduction

Bladder cancer is a widely diffused life-threatening risk for people in between 65 and 84 years of age, with men being targeted two to three times more than women [1]. In Italy, it is the fourth most common cancer in men (12%) and the fifth most common in the total population (8%), with 5-year survival estimated to be around 79% (http://www.salute.gov.it, 2019). Urinary cytology (UC) is an essential screening test in the detection of urinary tract cancers, most notably urothelial carcinomas [2]. Its main purpose is the surveillance and detection of urothelial neoplasms, with its strength being its specificity for the detection of high-grade carcinomas. In particular, today the examination of UT specimens in the cytopathology laboratory is typically used to screen for urothelial neoplasms in two populations: patients with new-onset and patients with a history of urothelial neoplasia, as urothelial carcinomas have high recurrence rates [3]. UC samples constitute a significant percentage of daily nongynecologic cases in any cytopathology laboratory and are one of the most difficult specimens that pathologists encounter [4].

As a result, trained clinicians have to analyze a very large number of UC samples daily, a process which is generally considered complex, time-consuming, and prone to strong intervariability. Because of this, a large amount of work has gone into the definition of precise criteria and methods to analyze UC samples and maximize their cost-effectiveness. Among them, the Paris System for Reporting Urinary Cytology (PSRUC) is currently the most successful categorization [5, 6]. While the categorization is considered efficient in practice [7], interpretation of UC images is still limited by a certain degree of subjectivity, large variations in interpretations, eye fatigue, and, most notably, time requirements, and the field could highly benefit from more effective support tools for partially automating, e.g., the diagnosis of easy, high-grade carcinomas.

In cytopathology, the combination of image analysis and deep learning could be the key to reduce the factors that can cause diagnostic errors, including the great variability of morphological features in the sample, the similarity between normal and suspicious forms, morphological alterations in the inflammatory context, and the difficulty of interpreting cellular alterations in case of inexperience. While the use of neural networks in cytopathology dates back at least to 1998 [8], recent progress in deep learning promises to provide more effective support tools in healthcare [9], with deep neural networks having obtained numerous high-profile successes ranging from diabetic retinopathy [10] to chest radiography and detection of skin cancer in dermatology [11]. Support tools for clinicians with high accuracy and sensitivity promise to significantly increase the cost-effectiveness of medical analyses in multiple fields, including cytology [12]. Still, multiple constraints and challenges need to be faced in order to make deep learning a suitable UC tool in support of clinicians, as described next.

### 1.1. Contributions of the Paper

This paper explores the usefulness of deep convolutional neural networks (CNNs) in the context of automatic detection of urothelial cancer cells from UC screenings. While a small number of preliminary works have explored similar ideas (see in particular the overview of related literature in Deep Networks for Medical Imaging), we identify a pair of shortcomings in past literature that we use as objectives when building the proposed architecture.

#### 1.1.1. Objective 1: Accuracy in the Small-to-Medium Data Regime

A standard pipeline for applying CNNs to medical imaging (shared by most prior works) is to leverage deep architectures originally designed for large-scale object recognition (e.g., the VGG, Inception, or ResNet families of models) and their pretrained weights originated from one or more real-world datasets [13]. We argue that this is suboptimal in our domain, where most datasets are relatively small in magnitude. To this end, we leverage recent work in multiexit deep networks (see Multioutput Deep Networks) to design a model that is more data-efficient in the regime under consideration. The basic idea is to endow a simple CNN with multiple auxiliary classifiers, which are able to process and predict a label at multiple scales and whose predictions are then adaptively combined during training, as depicted later on in Figure 1.

#### 1.1.2. Objective 2: Strong Calibration

Calibration refers to the match between the confidence of a model and the actual likelihood of the corresponding event in the ground truth data. Recent work has shown that deep CNNs tend to be poorly calibrated and overconfident on a number of examples [14]. In the medical domain, for systems that are used in support to the clinician, this is a problem insofar as a poorly calibrated confidence level cannot be used in a proper risk assessment procedure [15]. To this end, we explore two techniques to drastically improve the calibration of our model: training with a focal loss instead of the standard cross-entropy loss [16] and performing a posttraining calibration using temperature scaling [14].

To evaluate the proposed model, we collect a novel UC dataset with a retrospective study design on 60 patients, which we manually grade according to the PSRUC guidelines in normal and abnormal cells. The data collection and preprocessing pipelines are detailed next in Data Collection. In our experimental section, we show on our UC dataset and on a benchmark cell classification dataset that our multiexit, calibrated deep CNN strongly outperforms a baseline CNN both in terms of accuracy and in terms of calibration in all scenarios that we considered.

### 1.2. Organization of the Paper

The paper is structured as follows. In Related Works, we provide an overview of related works. Materials and Methods describes our proposed approach, both in terms of problem setup and model architecture (i.e., multiexit deep networks) and in terms of the steps we consider to calibrate the overall model. Data Collection details the procedure we followed to collect our UC dataset. Finally, Experimental Results provides a thorough experimental evaluation of the model, and we conclude in Conclusions with some final remarks.

## 2. Related Works

We organize our review of related works in three sections. In Deep Networks for Medical Imaging, we provide an overview on the application of CNNs to the medical domain and to urinary cytopathology in particular. In Calibrating Deep Networks, we overview recent work on evaluating the calibration of modern deep networks and improving their calibration during and after training. Finally, in Multioutput Deep Networks, we describe the reference literature for the field of multiexit deep networks.

### 2.1. Deep Networks for Medical Imaging

The interest in applying deep learning to healthcare stems from the large successes obtained by convolutional architectures on standard image classification benchmarks, such as ImageNet [17]. In the last years, CNNs have obtained several high-profile results in a variety of medical fields, ranging from classification of skin cancer in dermatology [11] to detecting diabetic retinopathy [10]. Further interest has been gained with the emergence of powerful methods for performing automatic segmentation of 2D [18] and 3D [19] biomedical data and for exploiting heterogeneous sources of information [20]. We refer the interested reader to specific surveys [12, 21–24] for an overview of CNN applications in medical histology and cytology. In the context of urinary cytopathology, a number of works [4, 25, 26] have shown promising preliminary results in automatically detecting carcinomas from urinary imaging. All of them, however, have focused on using out-of-the-box CNNs that are fine-tuned to the medical domain, while in this paper we design a more sophisticated architecture based on the two objectives described in Introduction.

### 2.2. Calibrating Deep Networks

Roughly, a calibrated network outputs confidences that are in line with the actual likelihood of the event, which is fundamental for a realistic risk assessment in a medical domain [15]. For neural networks, small models are generally well calibrated [3], while [14] was the first to observe that this rapidly degenerates in deeper architectures. Methods to recalibrate a binary classification model after training include histogram binning [27], isotonic regression [28], and Platt scaling [29]. Most of these methods can also be adapted to multiclass or regression scenarios. In particular, an extension of Platt scaling called temperature scaling [14] has become a de facto standard in deep networks, thanks to the possibility of improving the calibration at no cost in terms of accuracy. Temperature scaling is also widely used whenever the unnormalized probabilities of a network need to be smoothed, such as in knowledge distillation [30] and semisupervised learning [31]. Alternatively, it is possible to design proxy formulations for the calibration error [16] to be included inside the training process. Recently, [16] advocated for improving calibration by exploiting the so-called focal loss [32], which can be seen as training on a regularized criterion that increases the entropy of the predictions. In this work, we combine the focal loss with a posttraining calibration strategy to achieve a maximally calibrated model.

### 2.3. Multioutput Deep Networks

Before the introduction of batch normalization and residual connections, having several auxiliary classifiers at intermediate points in an architecture, to facilitate the flow of the gradient to early layers, was a common practice, e.g., in the Inception family of models [33]. However, these were removed afterwards, and only the last layer was used for predictions. Deeply supervised nets [34] were one of the earliest works to consider multiple exits to actually boost the accuracy of the model, especially in low-regime scenarios. A number of similar variants were proposed over the years, including BranchyNet [35], IDK Cascades [36], Adaptive Early Exit Networks [37], Deep Cascade Learning [38], and anytime predictions [39]. Part of these works is motivated by the possibility of training these architectures layer-wise (e.g., [38, 40, 41]). Another common thread is the idea of selecting an adaptive depth of the network independently for every input, which accelerates inference and can be beneficial especially in an edge context [35, 37]. Multiexit architectures also introduce challenges that are beyond the scope of this work, such as selecting the proper exit for each input [42]. By contrast, we adaptively combine all the exits in the proposed model with an additional linear layer, which is trained by backpropagation. Along this line, [43] considers soft combining all the outputs with an additional gating network. A tangential problem is selecting where to place the early exits [44, 45], which is a combinatorial problem of extreme importance whenever one faces energy and/or power constraints in IoT environments. For a more complete survey on the topic of multiexit neural networks, we refer the interested readers to [43].

## 3. Materials and Methods

### 3.1. Problem Setup

Denote by *x* a generic input image to the classification system. In this paper, the input is a fixed-size *H* × *W* × 3 crop of the original medical scan (in particular, *H* = *W* = 128 in the experimental section). The task is to train a suitable classification model *f*(*x*) that can diagnose the input image into *C* distinct classes, e.g., describing the type of cancerous cells present in the cropped portion of the image. Most deep learning models define *f* as the composition of *L* differentiable operations *f* = *f*^*L*^∘*f*^*L*−1^∘⋯∘*f*^1^, which can be either convolutional mappings, pointwise nonlinearities, pooling layers, batch normalization, or several others [46]. For example, a convolutional block is defined as

(1) $$\begin{array}{c} h^{i+1}=\phi \left(w★h^{i}\right), \end{array}$$

where *h*_*i*_ is the activation map from the previous layer, ★ denotes cross-correlation with the set of trainable weights *w*, and *ϕ* is a nonlinearity, typically ReLU (i.e., *ϕ*(*s*) = max(0, *s*)). Without loss of generality, the last operation of the network is always assumed to include a softmax normalization, in order to provide a suitably scaled probability distribution in output.

Given a set of *N* input-output examples {*x*_*i*_, *y*_*i*_}_*i*=1_^*N*^, with *y*_*i*_ being the index of the class for the *i*-th input, the model *f* is trained by minimizing a per-example cost to maximize its training accuracy:

(2) $$\begin{array}{c} L=\frac{1}{N}\overset{N}{\underset{i=1}{\sum }}\;l\left(y_{i},f\left(x_{i}\right)\right), \end{array}$$

where *l* is generally chosen as the cross-entropy loss:

(3) $$\begin{array}{c} l\left(y,f\left(x\right)\right)=-\underset{c}{\sum }\;I\left(y,c\right)\log\left(f_{c}\left(x\right)\right). \end{array}$$

with *f*_*c*_(*x*) denoting the probability assigned by the network to class *c* (the *c*-th value of the output vector), and *𝕀*(*a*, *b*) is an indicator function whose value is 1 whenever *a* and *b* are the same; otherwise, 0. Equation (2) can be optimized efficiently by performing stochastic optimization on minibatches of the full dataset.

Note that the output $\hat{p}=f\left(x\right)$ of the network provides a probability over classes, from which a prediction is generally made as $\hat{y}=\underset{c}{\text{argmax}}\left\{\hat{p}\right\}$. Then, we say that a model is calibrated whenever [14]

(4) $$\begin{array}{c} \mathbb{P}\left(\hat{y}=y\;\;|\;\;\hat{p}=p\right)=p,\;\forall p\in \left[0,1\right]. \end{array}$$

Similarly, we can define a calibration error (CE) that our model is incurring as

(5) $$\begin{array}{c} \text{CE}=E_{\hat{p}}\left[\;|\;\mathbb{P}\left(\hat{y}=y\;\;|\;\;\hat{p}=p\right)-p\;|\;\right]. \end{array}$$

In practice, both (4) and (5) need to be estimated from the data. The aim of this paper is to obtain a classification model for UC screening images which has simultaneously a high accuracy and a low calibration error, as described next.

### 3.2. Architecture

As a first point, in this paper, we propose to leverage the framework of multioutput models [43] to provide a more data-efficient model in the case in which *N* is in the small-to-medium range, which is common in medical applications. The general idea is to add a number of auxiliary classifiers departing from a set of middle points of *f*, such that the combined accuracy of all classifiers can improve over the accuracy of *f* alone. In this setup, we call *f* the backbone network, while we refer to each auxiliary classifier as an early exit.

More formally, denote by *𝒞* ⊂ {1, ⋯, *L*} a subset of layers of *f* after which we plan to insert an auxiliary classifier. While the choice of the optimal *𝒞* is in general a combinatorial problem [43], we consider here a simplified scenario wherein an early exit is added after each “macroblock” of *f*. All common deep learning models, such as residual networks [46], easily provide a way of identifying such macroblocks. For each *i* ∈ *𝒞*, we can obtain an early prediction as

(6) $$\begin{array}{c} {\overset{\wedge }{f}}^{i}\left(x\right)=c^{i}\left(h^{i}\right), \end{array}$$

where *h*^*i*^ = *f*^*i*^(*f*^*i*−1^(⋯*f*^1^(*x*))) is the intermediate output of *f* up to layer *i* and *c*^*i*^ is the auxiliary classifier. Auxiliary classifiers *c*^*i*^ are chosen as small classification models in order to introduce a negligible overhead in terms of computation and/or number of parameters (e.g., a single linear layer). Without loss of generality, we assume that *L* − 1 ∈ *𝒞*, so that the original output of the network is included among the early exits (slightly simplifying the notation to follow).

By denoting by *E* the number of early exits of the resulting model (*E* = ∣*𝒞*∣), the set ${\left\{{\overset{\wedge }{f}}^{i}\left(x\right)\right\}}_{i\in 𝒞}$ provides *E* possible classifications of the original image *x* (the original classification of the backbone plus *E* − 1 early exits). A relatively open problem in the field of multioutput NNs is how to properly select early exits for each input sample, in order to, e.g., balance the accuracy with respect to a computational budget [43]. In this paper, because our main aim is to boost the accuracy in a small-data regime, we propose a simple extension of the ideas in [43] to perform an ensemble of all outputs. In particular, denote by **f**(*x*) the vector concatenation of all early exits; the final decision of the model is taken by adding an additional linear layer:

(7) $$\begin{array}{c} f\left(x\right)=\text{softmax}\left(w^{T}f\left(x\right)\right), \end{array}$$

where **w** ∈ ℝ^*E*^ is a set of trainable coefficients to balance the contribution of each early exit (an alternative to (7) that did not provide significant gains in our experimental evaluation is to stack the classification vectors depth-wise and apply a set of 1 × 1 1D convolutions on top of them). The entire model can be differentiated and trained end-to-end.

An example with VGG-16 [17] as the backbone and five early exits is provided in Figure 1. In the figure, a “VGG block” corresponds to the original definition of blocks from [17], i.e., a sequence of 1 or more convolutive layers, followed by a max-pooling operation. Practically, we insert an early exit after every pooling layer. Exit 6 corresponds to the original exit from the backbone, while exit 7 is the combined output from (7), which is used for predictions (in this configuration, exit 5 is similar to exit 6 (a single linear projection applied on top of the last VGG block), but the parameters of the two linear projections are different. In a preliminary experimental evaluation, we have found a decrease in performance when removing exit 5).

We can also extend the cost function *l* to provide a more comprehensive error signal to the network by adding a loss term for each early exit for a single input as

(8) $$\begin{array}{c} \tilde{l}\left(y,f\left(x\right)\right)=\alpha l\left(y,f\left(x\right)\right)+\beta \left[\underset{i\in C}{\sum }\;l\left(y,{\overset{\wedge }{f}}^{i}\left(x\right)\right)\right], \end{array}$$

where *α* and *β* are two nonnegative real values that balance, respectively, the loss contribution from the combined output and the loss contributions from each of the early exits (including the original output of the backbone). Setting *α* = 0 (i.e., removing the combined output) recovers the deeply supervised model from [34]. Alternatively, setting decreasing rates for each loss term can help in rebalancing the gradient variance [39].

### 3.3. Model Calibration

The architecture described in the previous section helps in maximally exploiting the training information from the training dataset, by adaptively combining information at different scales in the network, as long as it propagates different types of error signals during the backpropagation phase. In this section, we consider the second objective from Introduction, i.e., the design of a maximally calibrated model. In particular, we speculate that the multiexit design can exacerbate the miscalibration problem discussed in Introduction. For this reason, apart from its importance in the context of medical risk assessement, calibration can also potentially improve the overall performance, as evidenced in the experimental section.

We consider a two-level calibration procedure, by (i) modifying suitably the loss function and (ii) applying a further posttraining calibration operation on the (combined) output of the network. For the former, we leverage the ideas from [16], and we substitute the classical cross-entropy loss in (2) and (8) with the more calibrated focal loss:

(9) $$\begin{array}{c} l\left(y,f\left(x\right)\right)=\underset{c}{\sum }\;I\left(y,c\right){\left(1-f_{c}\left(x\right)\right)}^{\gamma }\log\left(f_{c}\left(x\right)\right), \end{array}$$

where *γ* is a hyperparameter that is optimized on the validation set. An informal explanation for the performance of the focal loss is that it tends to favour points which have a low confidence, thus reducing the amount of overfitting on points either correctly predicted or wrongly predicted with strong confidence from the model [16]. In fact, it can be shown that while the cross-entropy is maximizing an upper bound on the Kullback-Leibler divergence $\text{KL}\left(\hat{p}\|p\right)$ between the predicted distribution $\hat{p}$ and the true one, the focal loss is maximizing a regularized upper bound [16]:

(10) $$\begin{array}{c} \text{KL}\left(\hat{p}\left\|p\right.\right)-\gamma ℍ\left[\hat{p}\right], \end{array}$$

where $ℍ\left[\hat{p}\right]$ denotes the entropy of the predicted distribution $\hat{p}$. We refer to [14, 32] for a more complete discussion on the properties of the focal loss.

To further improve the calibration strength of the model, we combine training on the focal loss to a postcalibration temperature scaling (TS) procedure [14]. Denoting by *t* = **w**^*T*^**f**(*x*) the combined output in (7) *before* the softmax, we replace after training the softmax with a scaled version of it:

(11) $$\begin{array}{c} {\tilde{f}}_{c}\left(x\right)=\frac{\exp\left(t_{c}/T\right)}{\sum_{j}\;\exp\left(t_{j}/T\right)}, \end{array}$$

where *T* is a separate hyperparameter, called temperature, that we optimize by minimizing the mean cross-entropy on the validation set (we have found no advantage in optimizing the temperature parameter directly on the focal loss over the validation set). TS has the advantage of slightly improving the calibration of the model, at no cost with respect to the accuracy, since the relative order of the predicted probabilities is not modified.

### 3.4. Data Collection

In order to evaluate the proposed architecture, we collect a novel UC dataset for testing the model. To this end, we take into consideration a retrospective study design on a dataset composed of images representing bladder tissue slides of 60 patients. Within the last 2 years, we collected material from the archive of the Cytopathology Laboratory Unit hosted in the Sant'Andrea Hospital from the Sapienza University of Rome, using the laboratory's electronic record system. Archived and well-preserved slides of urinary cytology with good material were chosen for the purpose of the study. All samples were prepared with conventional systems and stained with the Papanicolaou procedure. A digital still camera DP27 (Olympus) with a ×40 objective lens attached to a microscope BX45 (Olympus) was used to take the pictures focusing on the areas of interest in the smear. Criteria for inclusion in the dataset included having cells in monolayer arrangement that were well preserved and the exclusion of areas with excess of red blood cells, debris, and inflammation cells.

An expert cytopathologist reviewed all sets of achieved urine slides and manually identified representative categories of cells. The Paris system criteria [6] were used to classify urothelial cells. From this procedure, we obtained 274 images of urothelial normal cells and 416 abnormal cells. Among abnormal cells, we included atypical cells wherein the nuclear cytoplasmatic ratio was greater than 0.5 and when criteria such as nuclear hyperchromasia or irregular chromatin were detected. Suspicious cells were selected if the nuclear cytoplasmatic ratio was greater than 0.7 (i.e., associated with hyperchromasia, chromatin, and nuclear irregularity). Finally, we included high-grade urothelial cells with hyperchromasia, irregular nuclear contours, and coarse chromatin. The UC slides were prepared similarly using conventional systems and stained as described above. We show in Figures 2 and 3 a few representative examples from both classes.

### 3.5. Data Preprocessing

Because of the size of our dataset, we have the necessity of increasing it by applying some image preprocessing and data augmentation procedures. For this purpose, we follow the pipeline from [47], where the cytological images are initially cropped in 4 parts from the center point, obtaining four separate cell images from each original image in the dataset. We then randomly partition the dataset using 60% of the patients for training, 20% of the patients for validation (i.e., selection of all hyperparameters of the models), and the remaining 20% for testing. Performing the split at the level of each patient ensures that images (or crops) belonging to a single patient are all assigned to either training, validation, or test. For the training part only, we followed an additional data augmentation procedure and included, for each image, the corresponding rotation by 90°, 180°, and 270°. No additional preprocessing was performed on the data, in order to focus on the impact of the choice of the architecture and training strategies. Some additional statistics on the dataset are provided later on in Table 1.

## 4. Experimental Results

### 4.1. Experimental Setup

We evaluate the proposed multiexit, calibrated architecture from Materials and Methods on the UC dataset described in Data Collection. For completeness of evaluation, we also consider a separate benchmark dataset, the BCCD dataset of blood cell classification [48] (https://github.com/Shenggan/BCCD_Dataset). The BCCD dataset contains approximately 12,500 images of cells in four different classes, namely, eosinophil, lymphocyte, monocyte, and neutrophil. We consider this benchmark dataset in its original multiclass formulation and a binary formulation where we group all cells into granulocytes (neutrophils and eosinophils) and agranulocytes (lymphocytes and monocytes). We denote this last dataset as B-BBCD. Some general statistics about the three datasets that we consider, in terms of the number of classes and images in each set, are given in Table 1.

Apart from the standard accuracy on the test set, we are also interested in evaluating the overall calibration of the models, for which we follow the standard protocol of binning the output [14]. Specifically, we divide the interval of predictions into *M* = 10 equispaced bins, each of size 1/*M*. We denote by *ℬ*_*m*_ the indexes of points in the test set falling into the *m*-th bin and by *B*_*m*_ the corresponding cardinality (i.e., *B*_*m*_ = ∣*ℬ*_*m*_∣. We define the average accuracy over a bin as

(12) $$\begin{array}{c} \text{acc}\left(B_{m}\right)=\frac{1}{B_{m}}\underset{i\in B_{m}}{\sum }\;I\left({\hat{y}}_{i},y_{i}\right). \end{array}$$

Similarly, we can define the average confidence of the network on the bin as

(13) $$\begin{array}{c} \text{conf}\left(B_{m}\right)=\frac{1}{B_{m}}\underset{i\in B_{m}}{\sum }\;{\hat{p}}_{i}. \end{array}$$

From these, we can compute the expected calibration error (ECE), which is an approximation of (5) over the bins, as

(14) $$\begin{array}{c} \text{ECE}=\overset{M}{\underset{i=1}{\sum }}\;\frac{B_{m}}{N}\left|\text{acc}\left(B_{m}\right)-\text{conf}\left(B_{m}\right)\right|. \end{array}$$

We will use the ECE over the test set to evaluate the calibration of all models.

Our baseline model is VGG-16, a relatively common model in the context of medical imaging. We note that our main aim in the section is to evaluate the improvements in accuracy and calibration of our calibrated, multiexit model, which should be consistent over every choice of the backbone (we return on this point in the conclusive section). The VGG family provides a simple way of subdividing the main backbone into a number of blocks, which are identified by the presence of max-pooling operations [33]. In particular, we include 5 early exits into the model, each one composed of a flattening operation and a linear classifier. The overall architecture is described in Figure 1. To evaluate the impact of our proposals, we consider four variants for each architecture, by training with the cross-entropy loss or the focal loss and by performing temperature scaling after training or not. This gives us a total of eight variants. We train every variant with the Adam optimizer with a learning rate of 10^−3^ over minibatches of 32 images. Each experiment is averaged over 5 independent runs. All hyperparameters are optimized on the validation set.

### 4.2. Results and Discussion

Average results, in terms of test accuracy and test ECE, are provided in Table 2. As a first conclusion, we note that the standard CNN setup (no early exits, trained with a cross-entropy loss) has relatively poor performance in all scenarios that we consider, either by looking at the accuracy of the predictions and by looking at the average calibration, highlighting the two objectives we set up in Introduction. Simply performing a TS operation (second row of Table 2) can improve the ECE in two out of three cases, while maintaining a constant accuracy (by definition). The gain in ECE, however, is not guaranteed, and in the BBCD dataset, the average ECE only improves from 5.83% to 4.84%. Next, training a standard model with the focal loss, as advised in [14], can improve both the accuracy and the ECE in all scenarios. The improvement in ECE, however, is not consistent, in particular in the B-BBCD case, where the average calibration error only improves from 3.57% to 3.11%. Combining the focal loss with a posttraining TS provides a model that is generally well calibrated and slightly more performing than the standard one trained with a cross-entropy loss.

Importantly, our proposed multiexit model achieves significant improvements in accuracy over the baselines in all scenarios. In particular, when training with the cross-entropy loss, we improve over the baseline model by 2.53, 2.84, and 6 percentage points on the three datasets, respectively. Similarly, when training with the focal loss, we improve over the baseline models by 2.83, 2.32, and 6.54 percentage points, respectively. When considering the calibration of the models, we see from Table 2 that including the auxiliary classifiers generally worsens the ECE of the models. We conjecture, and we evaluate later on, that this is due to a poorer calibration of the first early exits in the models, which in general are only able to successfully predict a small number of simple examples [43]. While TS alone provides a good improvement over the ECE of the models, the best configuration (in terms of both test accuracy and test ECE) is always our proposed model combining multiexits, focal loss, and TS. In particular, we achieve the second-best ECE in the UC and B-BBCD cases and a significantly lower ECE in the BBCD case. Thus, we conclude that our proposed approach is a good proposal for satisfying the two objectives from Introduction in the case of medical imaging, especially UC screening.

### 4.3. Analysis of Calibration

To further evaluate the calibration of the models, we make use of reliability diagrams [14], a simple visual aid for understanding whether a model is calibrated and where it is making the most mistakes. In particular, in a reliability diagram, we plot the average confidence for each bin (the same bins we use to compute the ECE), highlighting with a red colour the gap with respect to a perfectly calibrated model, shown on the diagonal (i.e., a model for which (4) holds). We plot the reliability diagrams for the UC dataset (the one we are most concerned with) in Figure 4 for the models without TS and in Figure 5 for the models after performing TS. Like what we noted in the previous section, in the absence of TS, the standard model trained with the focal loss is the most calibrated, although it tends to be either overconfident or underconfident for the low-confidence regions, possibly because of the unbalance in the two classes in the dataset. For the models with TS, most variants are generally well calibrated, although the standard model with focal loss and the proposed model with the focal loss are the most calibrated, as also evidenced by the ECE in Table 2. Note, in particular, that while the former obtains a better ECE in Table 2, the reliability diagram provides a more comprehensive overview of the calibration of the model, showing that the latter is generally more behaved in low-confidence regions.

To provide even more insights, we consider a second common visual tool for evaluating the calibration of a model, called the confidence histograms, in Figure 6. The confidence histogram is a histogram of the model confidence on its most probable prediction, plotted alongside the average accuracy and confidence (using yellow and red dashed bars, respectively). The match between the two vertical lines provides a visual representation of the calibration. In particular, focusing our attention on Figure 6(c), we see that the reason for the low ECE exhibited by the multiexit architecture with the focal loss is the presence of a number of predictions made with a medium level of confidence, a region in which the model is significantly less calibrated (e.g., compare this with Figure 4(d)). Temperature scaling is able to reverse this behaviour by smoothing out these predictions, providing a calibration histogram in line with its other calibrated variants (e.g., Figure 6(b)).

Finally, we conclude by analyzing the average test accuracy and ECE for each early exit individually, focusing on the model trained with the cross-entropy loss on the UC dataset (results are similar for the other scenarios and are omitted for brevity). While these early exits are never used directly for the prediction (which is only obtained by the adaptive combination from (7)), analyzing their output in isolation provides some interesting information on the behaviour of the model. We show this in Figure 7, where the *x*-axis indicates the index of the early exit, with exit 6 being the original exit of the model (see Figure 1). We visualize the behaviour in both the presence and absence of temperature scaling. We already stated earlier that it is a known fact that the first early exits, when taken in isolation, have very poor test accuracy [43]. Here, we note that they also tend to have a correspondingly poor calibration, as shown in Figure 7(b). TS is able to uniform both the accuracy and the calibration of the exits to an extremely strong degree, thus contributing to an excellent trade-off between accuracy and calibration. In fact, we hypothesize that calibration is a fundamental topic for multiexit networks, and a further study in this context could provide valuable improvements even beyond medical imaging.

For completeness, we visualize in Figure 8 the evolution of the loss for the standard model compared to the multiexit model on a representative execution of the algorithms.

## 5. Conclusions

In this paper, we showed that a combination of multiple early exits, training with focal loss, and further calibrating the output of the model with a temperature scaling procedure produces models that are significantly more accurate and calibrated than baseline CNN architectures on cell classification problems. In particular, we evaluate the model on a novel urinary cytology dataset collected with a retrospective study design on 60 patients.

This study has a number of future works that we plan to explore over the following months. First, we envision to extend our data collection pipeline to include a more fine-grained evaluation for the cell dataset in accordance with the PSRUC guidelines and possibly extend beyond pure classification to segmentation and detection tasks. Secondly, attention-based models are currently achieving state-of-the-art performance in a number of domains [49], and we plan on investigating whether this gain extends to scenarios in medical imaging, particularly by endowing the transformer architectures with a number of early exits as done in this work. Finally, we envision to evaluate the interplay between early exits, calibration, and interpretability of the resulting activation maps, which is another major challenge in the medical domain.

## Figures and Tables

**Figure 1:** Example of the proposed architecture using a VGG-16 as a backbone network and 5 early exits included after each max-pooling operation. Exit 6 is the original exit from the backbone, and exit 7 the combined output from (7).

**Figure 2:** Representative examples from the normal portion of the dataset.

**Figure 3:** Representative examples from the abnormal portion of the dataset (see the main text for a description of the data collection procedure).

**Figure 4:** Reliability diagrams for the variants without posttraining TS.

**Figure 5:** Reliability diagrams after performing TS on the diagrams of Figure 4.

**Figure 6:** Confidence histograms for the multiexit models trained on the UC dataset.

**Figure 7:** Accuracy and ECE for each early exit for the proposed model on the UC dataset.

**Figure 8:** Evolution of the loss of the standard and multiexit model on the UC dataset.

**Table 1:** Statistics of the three datasets in the experimental section. UC refers to the custom dataset whose data collection procedure is described in Data Collection.

Dataset	# classes	Training images	Validation images	Test images
UC	2	2616	872	872
B-BBCD	2	7509	2503	2503
BBCD	4	7509	2503	2503

**Table 2:** Results (in terms of test accuracy and test ECE) of all eight variants evaluated on the three datasets. TS refers to a posttraining temperature scaling operation, as described in Model Calibration.

			UC		B-BBCD		BBCD	
Architecture	Loss	TS	Acc.	ECE	Acc.	ECE	Acc.	ECE
Standard	Cross-entropy	No	86.60%	4.77%	82.25%	3.57%	78.00%	5.83%
		Yes	86.60%	1.28%	82.25%	1.15%	78.00%	4.84%
	Focal	No	87.07%	1.50%	84.75%	3.11%	78.50%	3.72%
		Yes	87.07%	1.11%	84.75%	1.63%	78.50%	3.45%

Multiexit	Cross-entropy	No	89.13%	3.23%	85.09%	7.91%	84.00%	10.97%
		Yes	89.13%	2.30%	85.09%	2.78%	84.00%	5.21%
	Focal	No	89.90%	8.99%	87.07%	5.76%	85.04%	7.76%
		Yes	89.90%	1.43%	87.07%	1.57%	85.04%	1.97%

## Data Availability

The datasets of images used to support the findings of this study are available from the corresponding author upon request.
